# Heavyweight Statistical Alignment to Guide Neural Translation

**DOI:** 10.1155/2022/6856567

**Published:** 2022-06-03

**Authors:** Thien Nguyen, Trang Nguyen

**Affiliations:** ^1^Natural Language Processing and Knowledge Discovery Laboratory, Faculty of Information Technology, Ton Duc Thang University, Ho Chi Minh City, Vietnam; ^2^Faculty of Information Technology, University of Science, Ho Chi Minh City, Vietnam; ^3^Vietnam National University, Ho Chi Minh City, Vietnam

## Abstract

Transformer neural models with multihead attentions outperform all existing translation models. Nevertheless, some features of traditional statistical models, such as prior alignment between source and target words, prove useful in training the state-of-the-art Transformer models. It has been reported that lightweight prior alignment can effectively guide a head in the multihead cross-attention sublayer responsible for the alignment of Transformer models. In this work, we make a step further by applying heavyweight prior alignments to guide all heads. Specifically, we use the weight of 0.5 for the alignment cost added to the token cost in formulating the overall cost of training a Transformer model, where the alignment cost is defined as the deviation of the attention probability from the prior alignments. Moreover, we increase the role of prior alignment, computing the attention probability by averaging all heads of the multihead attention sublayer within the penultimate layer of Transformer model. Experimental results on an English-Vietnamese translation task show that our proposed approach helps train superior Transformer-based translation models. Our Transformer model (25.71) outperforms the baseline model (21.34) by the large 4.37 BLEU. Case studies by native speakers on some translation results validate the machine judgment. The results so far encourage the use of heavyweight prior alignments to improve Transformer-based translation models. This work contributes to the literature on the machine translation, especially, for unpopular language pairs. Since the proposal in this work is language-independent, it can be applied to different language pairs, including Slavic languages.

## 1. Introduction

Machine translation is one of the most complicated and prominent applications of artificial intelligence. Given a sentence in a source language, translation systems return a sentence in a target language, maintaining the meaning of the source sentence. Machine translation has a long history from the very first time modern computers were introduced. From the late 80s, machine translation resurged due to IBM statistical machine translation models [1, 2]. IBM models are word-based with different levels of complexity, based on word translation, word reordering, word deletion, and insertion. Word-based statistical models have long gone outdated, but their by-products in the form of word alignments are still attracting considerable interest. While modern neural models are now dominant in translation tasks, statistical approaches are still seen as more effective ways to align words [3]. Word alignments are a relation from the set of positions of words in the source sentence to the set of positions of words in the target sentence [4, 5]. The relation is composed of tuples (*i*, *j*), where *i* indicates *i*-th source word and *j* points to *j*-th target word. Although word-based statistical models are able to produce understandable translations, they fail to take into account the relations between words in sentences. As a result, they cannot generate fluent translations. Word-based statistical models were later replaced by phrase-based statistical models [6–8], which use word phrases as atomic units instead of words. Constructing more fluent translations, phrase-based models dominated the world of machine translation for a long time after the era of word-based statistical models. Nevertheless, they still require word alignment for building the phrase table, which is their integral component. In turn, phrase-based statistical models were surpassed by modern neural translation models. The introduction of neural networks to machine translation transformed the field. Neural translation models refer to deep neural networks following the encoder-decoder architecture [9]. The encoder of the model encodes sequences of source units as sequences of vectors of real numbers called “embeddings” [10–12]. The decoder of the model predicts the sequences of target unit embeddings based on source unit embeddings. Representing translation units as numerical vectors in a space, neural translation models are capable to measuring distances between words, therefore producing smoother and more natural predictions. Despite the numerical nature of neural translation models, statistical word alignments continue to prove useful for training these models. Many authors [13–18] used statistical prior word alignments in training recurrent neural translation models [19–21]. Specifically, they supervise the attention mechanisms [22, 23] in these models, using statistical prior alignments as the gold reference. Attention mechanisms are the crucial part of the decoder of the model. When the decoder decodes a target word, the attention mechanism allows it to look up the right word in the source sentence. The authors showed that recurrent models guided by prior alignments outperform the baseline models in many translation tasks, including English ⟶ French, German ⟶ English, Chinese ⟶ English, and English ⟶ Romanian.

Recently, Transformer models [24, 25] have established themselves as the state-of-the-art models in machine translation, as well as in many other fields [26–30]. In spite of the fact that many models take turns to dominate the machine translation fields, word alignments are still there, still showing their usefulness, even in the most modern, state-of-the-art Transformer models. Nguyen et al. [31] use statistical word alignment to train a Vietnamese ⟶ English translation model. They reported a significant improvement in the translation quality of the model. Although the improvement was witnessed, we still wonder whether the further improvement can be made. In this work, we experiment different techniques to achieve our goal of further improving Transformer-based translation models.

The paper is divided into six sections. After the introduction section, we review the related works in the second section.  Section 3 describes how to apply heavyweight prior alignments for training Transformer-based translation models.  Section 4 presents the experiments of the proposed approach on an English ⟶ Vietnamese translation task.  Section 5 outlines the experimental results and discussion. Some conclusions from the work are drawn in the final section.

## 2. Related Works

In this section, we give a brief overview of the studies which provide foundations for our work on applying heavyweight prior word alignment for training Transformer-based translation models.

Transformer models [24, 25] are famous for their multihead attention mechanism, which greatly contributes to their dominance in the machine translation field. Instead of a single head attention mechanism as in the case of recurrent neural models, Transformer models divide the constituent queries, keys, and values into multiple subqueries, subkeys, and subvalues, respectively. The subqueries, subkeys, and subvalues then perform the corresponding single attention mechanisms called heads. Finally, the results of the heads are concatenated.

Garg et al. [3] revised the training procedure for Transformer models, so that they can learn to translate and align together. In addition to the translation cost, the authors applied an alignment cost of weight = 0.05 in formulating the training cost. Statistical prior alignments generated with Giza++ tool [4] were used to train the models. The authors proposed to use the statistical prior alignment for supervising an arbitrary head of the 8-head attention mechanism in the penultimate layer of the decoder. They reported the improved alignment quality and unchanged translation quality in rich-resource English ↔ German translation tasks.

Nguyen et al. [31] adapted the work of Garg et al. to their low-resource Vietnamese ⟶ English translation task, improving the way to prepare statistical prior alignments. Specifically, they fed lemmas in place of words to the fast_align tool [5] to create prior lemma alignments. The prior lemma alignments were then used to train word-to-word translation models. They used the statistical lemma alignment to guide the first head of 8-head attention mechanism in the fifth layer of Transformer model consisting of six layers. As proposed by Garg et al., Nguyen et al. applied a cost function composed of a lightweight word alignment component in training the Transformer models. They reported a substantial improvement in the translation quality of the models for their low-resource translation task. In this work, we apply the same approach to prepare prior alignment and training procedures as in Nguyen et al.'s study [31] to train the baseline Transformer model. Moreover, we make some modifications with the goal to get better translation models. First, we apply a heavyweight word alignment component in formulating the cost function to train Transformer models. By doing that, we increase the role of prior alignment in training the Transformer models. The increase was inspired by a previous work on using prior alignments to train recurrent translation models. Chen et al. [13] used different weights for prior alignments, but all of them are heavy compared to weight = 0.05 as in the works [3, 31]. We also propose to further increase the role of prior alignments by using them to guide all heads of the 8-head attention mechanism.

## 3. Heavyweight Prior Alignment for Training Transformer-Based Translation Models

In this section, we describe how we formulate the optimization criterion to train Transformer-based translation models, increasing the role of prior alignments.

Given a training set of *N* sentence pairs and their corresponding statistical prior word alignments, Transformer models are trained with an optimization criterion consisting of a translation cost and a heavy alignment cost of weight = 0.5. In total, the training cost is represented in

(1) $$\begin{array}{c} C=C_{1}+0.5C_{2}. \end{array}$$

In (1), *𝒞*_1_ denotes the overall translation cost measuring the mismatch between the predictions of the decoder of Transformer model and the reference translations. We use the target sentences in the training dataset as references. *𝒞*_1_ is aggregated for all *N* target sentences.

(2) $$\begin{array}{c} C_{1}=\overset{N}{\underset{n=1}{\sum }}c_{1}^{\left(n\right)}. \end{array}$$

We compute each single-sentence translation cost *c*_1_^(*n*)^, following Muller et al. [32]. The mathematical formula of the translation cost is presented in

(3) $$\begin{array}{c} c_{1}^{\left(n\right)}=-\overset{L_{n}}{\underset{i=1}{\sum }}\overset{\text{D}}{\underset{j=1}{\sum }}\left(t_{ij}^{\left(n\right)}\times \text{log}\left(p_{ij}^{\left(n\right)}\right)\right). \end{array}$$

In (3), *p*_*ij*_^(*n*)^ is the probability the decoder predicts the *i*-th word in the *n*-th target sentence as the *j*-th word in the dictionary of the training dataset. *t*_*ij*_^(*n*)^ is the probability showing the correct answer in the reference target sentence of length *L*_*n*_. D is the size of the dictionary.

As in the case of the translation cost, the overall alignment cost *𝒞*_2_ is the aggregation of the individual alignment cost from all *N* sentence pairs in the training dataset.

(4) $$\begin{array}{c} C_{2}=\overset{N}{\underset{n=1}{\sum }}c_{2}^{\left(n\right)}. \end{array}$$

An individual alignment cost for *n*-th sentence pairs is computed as the difference between the statistical prior alignments and the average probabilities of all heads of the 8-head attention mechanism in the fifth layer of Transformer model consisting of six layers.

(5) $$\begin{array}{c} c_{2}^{\left(n\right)}=-\overset{L_{n}}{\underset{i=1}{\sum }}\overset{{\text{K}}_{\text{n}}}{\underset{j=1}{\sum }}\left(a_{ij}^{\left(n\right)}\times \text{log}\left(\overset{8}{\underset{h=1}{\sum }}q_{ij}^{\left(hn\right)}\right)\right). \end{array}$$

In (5), *K*_*n*_ and *L*_*n*_ are the length of *n*-th source and target sentence, respectively. *q*_*ij*_^(*hn*)^ is the probability that the *h*-th head of the attention mechanism points to the *j*-th word in the *n*-th source sentence when the decoder generates *i*-th target word. *a*_*ij*_^(*n*)^ is the probability projected from the statistical prior alignments for the *n*-th sentence pairs. If the *i*-th target is aligned to the *j*-th source word, then *a*_*ij*_^(*n*)^ takes a high value (i.e., 0.9), otherwise, a small one (i.e., (0.1/*K*_*n*_).

## 4. Experiments

### 4.1. Materials

We performed experiments on three English-Vietnamese bilingual datasets provided by Nguyen et al. [31], who had done preprocessing steps on the raw EVWA Corpus [33]. We use the training and development datasets to train Transformer-based translation models. We evaluate the quality of the translation models with the testing dataset. These datasets have 42026, 1482, and 1527 sentence pairs, respectively. Each sentence in the datasets is composed of no more than 80 words. All words in the datasets are in their true-case form. The true-case form is the most probable form of a word, for example, the word “It” with the form “it.” Some basic statistics of the datasets are demonstrated in Table 1.

### 4.2. Experimental Setup

The script for the experiments is presented as a Colaboratory code published on the GitHub website at the address https://github.com/ThienCNguyen/CInN_2022.

In this work, we prepare three word-to-word Transformer-based translation models guided with statistical prior alignments. The alignments are lemma-to-lemma, constructed according to the procedure proposed by Nguyen et al. [31]. For alignment, a word is represented by a corresponding lemma. A lemma is the root form of inflected words, such as the lemma “love” which is the root form of words “loves,” “loved,” “love.” By lemmatization, we lessen the sparse data problem, thus increasing the quality of alignment. First, we prepare Vietnamese lemmas with VnCoreNLP tool [34] and English lemmas with Stanza tool [35]. Secondly, we create English-to-Vietnamese and Vietnamese-to-English alignments with the fast_align tool [5]. Finally, the alignments are then combined according to grow-diagonal heuristics [36]. The statistical lemma-to-lemma alignments are then used to train word-to-word Transformer-based translation models.

Following the works [3, 31], we use lightweight prior alignments of weight = 0.05 in the training cost to train the first Transformer model. The alignments guide the first head of the attention mechanism. We consider it as the baseline translation model (Transformer-L1) in this work. After that, we train the second Transformer model (Transformer-H1) with the heavyweight prior alignment of weight = 0.5, maintaining the guidance for only the first head. Finally, we train the third Transformer model (Transformer-HA) with heavyweight prior alignments guiding all heads of the attention mechanism of the model.

Except for the formulation of the training cost, all Transformer models have the same architecture and training procedure. Specifically, both the encoder and decoder of the model have six layers. The attention part of a layer contains eight heads. The feed-forward network in a layer is of 2048 dimensions. Embeddings of 512 dimensions are used for both the encoder and decoder. The dropout level of the models is 0.3. The models are trained with Adam optimizer [37] of *β* = (0.9, 0.98). We apply the 2*e*^−4^ learning rate. The training process of the models will be terminated if it reaches *e*^4^ steps of 3200 words, or the training cost is not improved by *e*^−4^. During the training process, we store the parameter values of a model after a completion of an epoch. To avoid the overfitting problem, we select the parameter values providing the best result in the separate development dataset.

We implement the Transformer models with open-source Fairseq Toolkit [38], written in high-performance library PyTorch [39]. We prefer Fairseq to other famous sequence modeling toolkits, such as OpenNMT [40, 41], because it is fast and extensible to our needs.

After we train the translation models, we feed English sentences of the testing dataset to them. The model searches the possible translations with beam size = 5. We compare the translations with the corresponding Vietnamese sentences of the testing dataset in terms of BLEU score [42]. The scores are calculated with multi-bleu.perl using the statistical machine translation toolkit Moses [43].

We also complement the automatic BLEU score with the judgment on the translation results by native speakers of the target language. The criterion of human judgment is the similarity in meaning between the target and the source sentence. As was done in the works [44–46], native speakers evaluate Vietnamese translation results from five English source sentences which are arbitrarily taken from the testing dataset. We only fix the length of the selected source sentences from 8 to 16 with step = 2 tokens.

## 5. Experimental Results and Discussion

Figures 1–3 show the change of costs over the training epochs for Transformer-L1, Transformer-H1, and Transformer-HA models, respectively. We studied three types of costs: training cost, constituent alignment cost, and development cost. For the all three models, the training cost and the alignment cost decrease over time. At the same time, the development cost first decreases and then increases, resulting in the lowest point. At the lowest point, we selected the parameter values for the model. The baseline Transformer-L1, Transformer-H1, and Transformer-HA models converged after 21, 23, and 30 training epochs, respectively. Comparing the lowest points, we found that the baseline model requires the least number of training epochs, while the Transformer-HA model uses the most, almost 50% more than the baseline model.

The result of automatic evaluation of the Transformer models is presented in Figure 4. They are BLEU scores of translations for the testing dataset. We found that the proposed heavyweight models provide better BLEU scores than the baseline lightweight Transformer-L1 model. In particular, the proposed Transformer-H1 and Transformer-HA models surprisingly improve the translation results by 2.52 and 4.37 BLEU, respectively. The relative improvements of 11.8% and 20.5% are unexpectedly good. The results prove that the role of statistical prior alignment for training the Transformer models is essential. The larger the role they play, the better translation Transformer models generate. Specifically, we increased the role of prior alignments in the training cost, and we successfully built a better Transformer-H1 model, compared with the baseline Transformer-L1 model. When we applied a heavy weight for prior alignments and made them guide all heads of the multihead attention mechanism, we created the Transformer-HA model providing the better improvement of 20.5%.

Experimental results also reveal that the slower the convergence time is, the better the translation model is. The baseline lightweight Transformer-L1, the proposed Transformer-H1, and Transformer-HA models, converging after 21, 23, and 30 training epochs, provide translation quality of 21.34, 23.86, and 25.71 BLEU, respectively.

While the automatic BLEU score is convenient for comparing translation results, especially from thousands of sentences, we are still interested in the translation quality from the point of view of translators. That is why we did limited case studies with some translation results. In this report, we present five case studies of translation quality evaluation.

Table 2 presents the translations from an English sentence of 8 tokens by the Transformer models. This case shows the superiority of the proposed Transformer-HA model over the other models. It successfully keeps the important keyword Alzheimer in the Vietnamese translation “An-dai-mơ.” In general, the meaning (How do people know if they have Alzheimer?) of the translation by the Transformer-HA model is similar to the source sentence. At the same time, the baseline Transformer-L1 and the proposed Transformer-H1 do not generate translations reflecting the meaning of the source sentence.

Table 3 shows the translations from an English sentence of 10 tokens by the Transformer models. In this case, both the proposed Transformer-H1 and Transformer-HA models provide good enough translation, while the baseline Transformer-L1 model fails to do it. The proposed models correctly translate the source phrase “over 65 years of age” into “trên 65 tuổi” (meaning: over 65 years old). Unfortunately, the baseline mistranslates the phrase into “đến 65 tuổi”(meaning: up to 65 years old).

Table 4 compares the translations from an English sentence of 12 tokens by the Transformer models. In this case, all models literally express themselves pretty well. They successfully translate most source words. However, the proposed Transformer-HA model proves to be the best. Although all three models give similar translation in terms of vocabulary, only the Transformer-HA provides a proper word order. Vietnamese is an analytic language, where word order plays a role in defining the meaning. The translation phrase “được điều trị lâu hơn” (meaning: be treated for longer) by the Transformer-HA model better reflects the meaning of the source sentence than its permutation “lâu hơn được điều trị” (meaning: longer before being treated) provided by the other models.

Table 5 displays the translation from an English sentence of 14 tokens by the Transformer models. In this case, all models provide good translations, reflecting the meaning of the source sentence. Nevertheless, we consider the translation by the proposed Transformer-HA model is the smoothest. The translation phrase “đã ngưng điều trị sớm” (meaning: prematurely stopped treatment) completely matches the reference “đã ngưng điều trị sớm,” while the corresponding translations “ngưng điều trị sớm hơn” (meaning: stop treatment earlier) by the baseline Transformer-L1 model and “dừng lại điều trị sớm” (meaning: stop treatment soon) by the Transformer-H1 model sound unnatural in Vietnamese.

Table 6 exhibits the translations from an English sentence of 16 tokens by the Transformer models. In this case, all models fail to translate the key source phrase “to keep an eye on,” as a result providing mistranslations. Except for that, all models successfully translate other parts of the source sentence. In terms of BLEU score, the translations are not bad at all. However, from the point of view of human translators, they do not reflect the meaning of the source sentence. It is the main reason BLEU score is accompanied by human judgment in our work.

In general, the limited human judgment actually confirms the automatic machine judgment with BLEU score. The proposed Transformer-H1 and Transformer-HA models outperform the baseline Transformer-L1 model; especially, the Transformer-HA model shows its superiority by being able to provide correct word order and translate rare key words. In addition, we notice that the performance of the models worsens when the length of source sentences increases. This limitation will be addressed in the future works.

## 6. Conclusions

In this work, we have raised the importance of prior alignment in training the English ⟶ Vietnamese Transformer-based translation models. Experimental results showed that translation models trained with heavyweight prior alignments provide a significantly better BLEU score than a strong baseline model. The baseline model is Transformer-based with lightweight prior alignment guiding the first head of the multihead attention mechanism. In addition, when we use heavyweight prior alignment to guide all heads of the multihead attention mechanism, we noticed even larger differences in BLEU scores between the baseline and the proposed models. Limited human evaluation of the translation quality actually validates the automatic machine judgment. We recorded the significant improvement in the translation quality of our proposed translation models over the baseline model.

Given the discovery in our work, we recommend heavyweight prior alignments to guide all heads of the multihead attention mechanism of the Transformer translation models. The training procedure may help generate better translation models for low-resource language pairs, such as English ⟶ Vietnamese.

## Figures and Tables

**Figure 1:** The cost of training the baseline Transformer-L1 model.

**Figure 2:** The cost of training the Transformer-H1 model.

**Figure 3:** The cost of training the Transformer-HA model.

**Figure 4:** BLEU scores of translation by the models.

**Table 1:** Some basic statistics of the datasets.

English-Vietnamese	Training	Development	Testing
Sentence pairs	42026	1482	1527
Average lengths	19.2–26.2	17.8–24.5	20.6–28.3
Words	806456–1099205	26315–36276	31513–43286
Dictionaries	36672–16441	4981–2720	6211–3462

**Table 2:** Translation from an English sentence of 8 tokens.

	Case study 1
English source	“How do people know they have Alzheimer?”
Vietnamese reference	“làm sao người ta biết mình mắc bệnh An-dai-mơ?”
Translation by Transformer-L1	“người ta biết họ đã làm thế nào?”
Translation by Transformer-H1	“làm thế nào cho người ta biết họ có bị đổ vỡ như thế nào?”
Translation by Transformer-HA	“làm thế nào mà mọi người biết có bị An-dai-mơ không?”

**Table 3:** Translation from an English sentence of 10 tokens.

	Case study 2
English source	“It usually affects people over 65 years of age.”
Vietnamese reference	“đối tượng thường mắc bệnh là người già trên 65 tuổi.”
Translation by Transformer-L1	“người ta thường ảnh hưởng đến 65 tuổi.”
Translation by Transformer-H1	“nó thường ảnh hưởng đến mọi người trên 65 tuổi.”
Translation by Transformer-HA	“nó thường xảy ra ở những người trên 65 tuổi.”

**Table 4:** Translation from an English sentence of 12 tokens.

	Case study 3
English source	“The longer patients were being treated, the more reported side effects.”
Vietnamese reference	“bệnh nhân nào được điều trị càng lâu thì chịu tác dụng phụ càng lớn.”
Translation by Transformer-L1	“bệnh nhân lâu hơn được điều trị, càng nhiều các tác dụng phụ hơn.”
Translation by Transformer-H1	“bệnh nhân lâu hơn được điều trị, báo cáo các tác dụng phụ hơn.”
Translation by Transformer-HA	“bệnh nhân còn được điều trị lâu hơn, theo báo cáo nhiều tác dụng phụ hơn.”

**Table 5:** Translation from an English sentence of 14 tokens.

	Case study 4
English source	“A UK charity said it was aware some women stopped their treatment early.”
Vietnamese reference	“hội từ thiện Anh quốc nói rằng họ biết một số phụ nữ đã ngưng điều trị sớm.”
Translation by Transformer-L1	“tổ chức từ thiện Anh cho biết họ nhận thức được một số phụ nữ ngưng điều trị sớm hơn.”
Translation by Transformer-H1	“tổ chức từ thiện Anh cho biết họ nhận thức được một số phụ nữ dừng lại điều trị sớm.”
Translation by Transformer-HA	“tổ chức từ thiện Anh cho biết họ nhận thức được một số phụ nữ đã ngưng điều trị sớm.”

**Table 6:** Translation from an English sentence of 16 tokens.

	Case study 5
English source	“Besides the overheating issues, here are several other problems to keep an eye on.”
Vietnamese reference	“bên cạnh các vấn đề nhiệt độ, ở đây còn một số vấn đề khác cần phải để mắt đến.”
Translation by Transformer-L1	“ngoài những vấn đề quá nóng, đây là một số vấn đề khác để giữ mắt.”
Translation by Transformer-H1	“ngoài các vấn đề quá nóng, dưới đây là một số vấn đề khác để giữ mắt lên.”
Translation by Transformer-HA	“ngoài các vấn đề quá nóng, dưới đây là một số vấn đề khác để giữ cho mắt.”

## Data Availability

The text data used to support the findings of this study are available from the corresponding author upon request.
